# Purification and characterization of novel isoforms of the polyphenol oxidase from *Malus domestica* fruit pulp

This article has been retracted.

**DOI:** 10.1371/journal.pone.0276041

**Published:** 2023-08-25

**Authors:** Naila Sajjad, M. Sheeraz Ahmad, Raja Tahir Mahmood, Muhammad Tariq, Muhammad Javaid Asad, Shamaila Irum, Anisa Andleeb, Abid Riaz, Dawood Ahmed

**Affiliations:** 1 University Institute of Biochemistry and Biotechnology (UIBB) & National Center of Industrial Biotechnology (NCffigIB) Pir Mehr Ali Shah, Arid Agriculture University, Rawalpindi, Pakistan; 2 Department of Biotechnology, Mirpur University of Science and Technology (MUST), Mirpur AJK, Pakistan; 3 Department of Zoology, University of Gujrat, Gujrat, Pakistan; 4 Department of Plant Pathology, Pir Mehr Ali Shah, Arid Agriculture University, Rawalpindi, Pakistan; 5 Department of Medical Laboratory Technology, University of Haripur, Haripur, KP, Pakistan; Government College University Faisalabad, PAKISTAN

## Abstract

Polyphenol oxidases (PPOs), belong to the group of oxidoreductases that are copper containing enzymes and are responsible for plant browning. PPOs are extensively distributed in plant kingdom and can oxidize wide range of aromatic compounds of industrial importance. The aim of this study was purification and characterization of PPO isoforms from the fruit pulp of Golden delicious apple. High performance liquid chromatography was used to purify the two novel isoforms of PPO and further their molecular weights (45 and 28 kDa) were determined using sodium dodecyl sulfate polyacrylamide gel electrophoresis. The purified isoforms have optimum pH (6.5), optimum temperature (40°C), the V_max_ (4.45 μM/min) and K_m_ (74.21 mM) with catechol substrate. The N-terminal microsequences of both PPO isoforms were determined using a pulse liquid protein sequencer and found to be AKITFHG (28 kDa) and APGGG (45 kDa). Polyphenol oxidases are efficiently used in the pharmaceutical, paper and pulp, textiles and food industries. Recently, the PPOs have been used for bioremediation and in the development of biosensors.

## 1. Introduction

Enzymatic browning observed in vegetables and fruits are natural processes that result in the significant loss of food quality including change in taste, color, flavor, and decrease nutritional value. Polyphenol oxidases (PPOs) are widely present in animals and plants, especially vegetables (mushroom, potatoes, eggplant, lettuces, melon and guava) and fruits (grape, apple, avocado, peach, mango, pear, apricot, and banana) [1]. PPOs are said to catalyze oxidation and reduction reactions that oxidize phenols and aromatic compounds to quinones which further catalyze non-enzymatic reactions to produce colored pigments and its active site consist of two copper atoms [2, 3]. PPOs catalyze two types of activities hydroxylation of monophenols by monophenolases and oxidation of diphenols by diphenolases involving their copper atoms. Three common types of PPOs are tyrosinase, catechol oxidase and laccase [4]. Initially, plant polyphenol oxidases are synthesized as pre-proteins which takes plastid transit peptides at amino terminal region that help to target the PPOs into thylakoid [5]. The disruption of cell membrane integrity in fruits and vegetables results in the phenolic substrates to move towards the enzyme and cause browning which decreases the acceptability of the food stuff and causes considerable economic loss in food processing industry [6, 7]. PPOs can be used for many beneficial purposes, in textile industry (decolorization and denim bleaching), food industry (increasing aroma and color of tea and coffee), preparation of hair dyes and skin lightning agents [8]. PPO reduces the sticking of a bacterium, *Streptococcus sobrinus*, which forms the oral cavity on the surface of tooth.

Polyphenolic compounds are extensively studied in literature due to their nutraceutical properties and having beneficial effect on human health in respect to antioxidant activity, anti-bactericidal, cardiovascular and anti-inflammatory response [9]. Recent studies on extra virgin olive oil and cocoa beans showed the presence of polyphenol oxidase rich nutrients and nutraceuticals in them, having antiplatelet and antioxidant activities. Furthermore, polyphenol oxidases have a significant function in preclinical and clinical diagnosis and it has a role in treating Parkinson’s disease [10] and also used as a biomarker for Vitiligo [11]. PPOs are also reported to reduce the risk of cardiovascular diseases especially in the regulation of cardiovascular risk factor (insulin sensitivity, blood pressure, downregulation of oxidative stress, serum cholesterol and platelet aggregation) and myocardial infarction [12]. Reported studies also confirm that the PPOs are used in the treatment of Alzheimer disease [13]. Polyphenol oxidases have a crucial function in defense mechanism of plants [14]. The polyphenol oxidase enzyme can be immobilized on many matrices like glass beads, carbon based [15], hydrogel, mesoporous silica materials, nafion membranes and organic sources such as chitosan [16].

The PPOs are coded by the family of genes having highly conserved multiple genes [17]. The sequence analysis by Edman degradation is the most accurate method that provides researchers the complete amino acid sequence information [18]. This process involve the chemical modification of the amino acid at N- terminal, its cleavage from the peptide and further cleaved labeled amino acids were identified using high performance liquid chromatography (HPLC) [19]. In the last century, PPOs were considered to be the most significant enzymes and their different isoforms have been identified from different plant sources with varying number and sizes [20]. The next decade is likely to see PPO as an important enzyme for industries due to its significant applications. Previous study has focused on its extraction and has isolated PPO isoforms from different apple varieties but neither work has been reported from Golden delicious apple, nor from pure fruit pulp [21, 22].

As apple is rich in phenolics so we designed our work to isolate, purify and characterize the polyphenol oxidase isoforms from Golden delicious apple fruit pulp. High performance liquid chromatography was used for enzyme purification. We have studied the optimum pH, temperature, metal ion effect and kinetics using the purified PPO. This study describes the new approach of amino acids sequencing of purified PPOs from the N-terminal region.

## 2. Materials and methods

### 2.1 Materials

The fresh Golden delicious apple (*Malus domestica*) fruit was used for PPO extraction. The polyphenol oxidase from the apple fruit pulp was extracted by using phosphate buffer (0.1M, pH 7). Proteins were precipitated using cold acetone followed by centrifugation. HPLC (Water 1525 Binary Pump) was used with superdex column and was performed in Case Western Reserve University, Ohio USA. NuPAGE Novex Bis**-**Tris Gels for SDS-PAGE in X Cell SureLock Mini Cell (USA) was used. Gel was transferred on Polyvinylidene diflouride membrane (PVDF) by western blotting (wet blotting). A sequencer (Pulse liquid, ABI Model 477A) with applied Biosystems’s computer program was used for amino terminal sequencing of proteins and was done in USA. All of the chemicals and reagents used in the given study were obtained from Sigma Aldrich USA.

### 2.2 Extraction and purification of polyphenol oxidase

Fresh apple fruits were cut into thin slices after peeling and crude polyphenol oxidase extracts were prepared after homogenization of the sliced fruit in blender for 5 min in sodium phosphate buffer (80g/0.1 M, pH 7). Centrifugation for 90 min at 8,000 rpm was done to collect the supernatant and stored at 4˚C for future experiments. The extraction was carried out following the method as described previously [23] with some modifications. Briefly, the PPO was precipitated from the crude extract using acetone precipitation (1.5 volumes cold acetone to 1 volume crude extract) and placed on continuous stirring at 4˚C for 8h Centrifugation at 8,000 rpm for 30 min was done and collected precipitates were dissolved in 10 mL phosphate buffer (0.1 M, pH 7). The method was used as described previously [24] with minor modifications. The standard chromatogram was obtained initially by injecting bovine serum albumin as a standard into the HPLC superdex column. One milliliter protein sample obtained after acetone precipitation was then injected. Each fraction having 3 mL volume was collected during each 24 min run after washing the column with phosphate buffer, 0.1 M (pH 7). All the collected fractions were tested to determine protein concentration [21] and PPO activity [25]. Polyphenol oxidase assay was performed using substrate (catechol) and active fractions having PPOs were used in further experiments [26].

### 2.3 SDS-PAGE

Standard protocol of NuPAGEBis-Tris Mini was used for SDS-PAGE using mini cell of X cell Sure Lock. The reducing agent and LDS sample buffer of NuPAGE was used to prepare the samples (100 μL). The samples were heated for 5–10 min before loading into the gel cassette wells. Gel running buffer (1X SDS) was prepared using MOPS SDS or 20X MES running buffer of NuPAGE (50 mL) and 950 mL deionized water. The gel cassette was then submerged into X cell sure lock and 1X running buffers were used to load the upper and lower buffer chambers. Electrophoresis was done at 200V for 35 min. After completion the gel was completed and stained in the staining solution containing 20 mL methanol, 20 mL stainer A, 55 mL deionized water and 5 mL stainer B [27].

### 2.4 Polyphenol oxidase activity measurements

PPO assay was performed from apple fruit pulp extract at all stages of purification using 960 μL of 0.1 M sodium phosphate buffer (7 pH) and 200 mM catechol solution (20 μL). The rate of reaction was studied after adding the enzyme solution (20 μL). Catechol was used as a substrate and spectrophotometer was used to read the absorbance at 420 nm (Thermo Scientific Evolution 60S) and enzyme unit was used to expressed the enzyme activity which is defined as the amount of enzyme that caused 0.001 changes in absorbance in 1 min. Enzyme assay was performed by the method as described by [28] with some modifications.

### 2.5 Characterization of polyphenol oxidase

The PPO activity was observed at optimum pH by adding buffers with varying pH (3–7) and polyphenol oxidase assay was performed using catechol substrate. The enzyme solutions were incubated at different temperatures (30°C—70°C for 15 min and adjusted at the given temperatures one by one for the optimization of temperature. The reaction rate was measured after adding the substrate solution and PPO activity was determined at room temperature after incubating the enzyme solution in the afore-mentioned temperatures. Metal ions play a vital role in biological functions of most of the enzymes. Those enzymes that catalyze oxidoreduction reactions mostly contain iron, molybdenum as well as copper. Various types of interactions occur among metals, substrate or inhibitors as well as enzyme proteins. In the current study metal ions (1mM) concentration of calcium, copper and potassium (CuSO_4_, KCl, CaCl_2_) were added in the enzyme solution and polyphenol oxidase activity was studied with catechol substrate. Michael-Menten constant (K_m_) for the polyphenol oxidase was determined and maximum rate of reaction (V_max_) was calculated by using lineweaver-Burk plot method [24].

### 2.6 Protein blotting

Proteins were transferred to the membrane for chemical characterization by using wet blotting. Polyvinylidene difluoride (PVDF) base membrane was used for N-terminal microsequencing and a membrane that can resist the chemicals of the sequencer was used. Whatman 3MM filter paper, blotting buffers, electrophoresed gel, blotting membrane, electroblotting equipment and electrophoresed gel were used. A standard method of wet blotting for transferring the gel to the membrane (PVDF) was used. Briefly, blotting buffer was added in a dish and the anode face of blotting cassette was placed in it. We put a sponge pad above the anodic face of the blotting cassette after inundation. The two pieces of Whatman 3 MM filter paper was placed on the sponge pad and rolled in such a way to remove all air bubbles in the next step. PVDF**-** blotting membrane was placed in the blotting buffer on top of the sandwich of blotting after dipping in methanol. The previously electrophoresed gel was kept on top side of the membrane used for blotting and the sponge pad was kept into the buffer and then on above side of gel. The cassette of blotting with cathode side up was placed on the top of the sponge pad and fastened tightly to the anode side. The blotting cassette was placed into the blotting tank filled with transfer buffer after removing from the dish of buffer and joined to the power supply at 500 mA for 2h.

### 2.7 Protein staining for N-terminal microsequencing

The blotting membrane was removed from the sandwich assembly and was placed for 2 min into a dish having coomassie brilliant blue staining solution (0.2% (w/v) with the following composition (methanol 45% v/v, acetic acid 10% v/v in deionized water) on a gentle shaker. Further the PVDF membrane was transferred in to the de-staining solution with constant shaking until pale color background appeared, washed with water (deionized) and air dried. A clean plastic bag was used to place the stained membrane for future use and pulse-liquid protein sequencer (ABI Model 477A) was used for N-terminal microsequencing. A razor blade was used to cut the polyvinylidene blot having proteins, washed with deionized water and further placed into the cartridge blot fixed on the protein sequencer. The cartridge design matched exactly according to its use with blotting membranes and it permits cross flow in vertical direction instead of the flow that occurs by using usual ABI sequencing cartridge. This layout has solved the problem of slow flowing due to small size of the Polyvinylidene difluoride base membrane that allow for the complete chemistry. The blot was dried inside the sequencer by using argon before performing Edman degradation.

### 2.8 Statistical analysis

Each experiment was done in triplicates and all the data for the studies of biochemical properties of PPOs were presented by means ± standard error using descriptive statistical methods and regression. The graphs were prepared using the graph pad prism software.

## 3. Results

### 3.1 Purification of PPOs

PPOs activity of Golden delicious apple fruit pulp crude extract (3.55 μM/min), acetone precipitation (3.06 μM/min) and HPLC (14.111 mg/mL) was determined. Total protein concentration of crude extract (18.228 mg/mL), acetone precipitation (14.111 mg/mL) and HPLC (0.843mg/mL) was also found. The specific activity of crude extract (0.19 U/mg), acetone precipitation (0.211 U/mg) and HPLC (1.17 U/mg) was calculated. The yield was taken to be crude extract (100%), acetone precipitation (86%) and HPLC (27%) and was purified to be 6.15 folds (Table 1). The enzyme activity of each fraction obtained through high performance liquid chromatography was observed by performing enzyme assay and PPO active fractions were collected at 12.835 min with 0.3 absorbance on spectrophotometer (Fig 1).

**Fig 1:** Elution profile of *Malus domestica* (Golden delicious apple) fruit pulp PPO isoforms obtained from HPLC. Superdex column was used at retention time (RT) 12.835 min with 0.3 absorbance on spectrophotometer. Time period (24 min) is plotted on horizontal axis and absorbance is plotted on vertical axis.

**Table 1:** Stepwise purification result of the fruit pulp of Golden delicious apple polyphenol oxidase.

Steps	Total Activity (μM/min)	Total Protein mg/mL	Specific Activity (U/mg)	Yield (%)	Purification (Folds)
**Crude Extract**	3.55	18.228	0.19	100	1
**Acetone Precipitation**	3.06	14.111	0.211	86	1.10
**HPLC**	0.99	0.843	1.17	27	6.15

### 3.2 SDS-PAGE

The purified PPOs in apple migrated as two active bands in the gel having 45kDa and 28kDa (Fig 2) which shows that enzyme is a dimer. Two active PPO isoforms were detected in Fig 2 that were compared with Lane 1 and 2 having molecular markers.

**Fig 2:** SDS-PAGE gel electrophoresis of the purified polyphenol oxidase isoforms from the fruit pulp of Golden delicious apple. Lane 1 & 2: molecular weight markers. Lane 3–5: apple PPO samples in triplicate. Gel is showing two active bands of PPO isoforms (28 and 45 kDa).

### 3.3 Optimum pH of apple PPO

In the enzyme active sites, the change in the ionization of prototropic groups affects the substrate binding, proper active site conformation and reaction catalysis. The decrease in stability of the substrate as well as irretrievable denaturation of protein as a pH function could affect the enzyme catalytic activity. The results showed that polyphenol oxidase activity was optimum at pH 6 and 6.5 (Fig 3). Figure showed that pH has strong effect on the activity of PPO purified from Golden delicious apple with catechol substrate and enzyme was also active at high pH but its activity start decreasing at highest pH.

**Fig 3:** pH optimization of polyphenol oxidase isoforms purified from the fruit pulp of Golden delicious apple. Each bar plot is showing the mean value of the polyphenol oxidase activity at varying pH (3–8). Error bars are representation of standard error (SE) of the data. Horizontal axis is showing phosphate buffer of varying pH and vertical axis is showing polyphenol oxidase activity at different pH is plotted on vertical axis. Graph is showing maximum activity of Golden delicious apple fruit pulp PPO at pH 6 to 7.

### 3.4 Optimum temperature of apple PPO

Temperature is one of the main factors that affect the PPO catalytic activity. At high temperature, enzymes lose 3-dimensional structure and denature. Temperature variations may change oxygen solubility; the most important factor that is required for the PPO to perform its catalytic function. The results showed the PPO activity from Golden delicious apple fruit pulp was greatest at 40°C and it was slightly less above that temperature (Fig 4). According to Fig 4, change in temperature also has considerable effect on PPO activity with catechol substrate. Enzyme was active and stable but its activity slightly starts decreasing due to enzyme denaturation at highest temperature.

**Fig 4:** Optimization of temperature of the purified isoforms of polyphenol oxidase purified from the fruit pulp of Golden delicious apple. Each bar plot is showing mean value of the polyphenol oxidase activity at varying temperatures (30°C-70°C). Error bars are representation of standard error (SE) of the data. Horizontal axis is showing the temperature in °C and vertical axis is showing the polyphenol oxidase activity. Graph is showing maximum activity of Golden delicious apple fruit pulp PPO isoforms at 40˚C.

### 3.5 Effect of metal ions on PPO

The neither increased nor decreased in the PPO activity was observed in the presence of KCl, CaCl_2_ but the addition of copper ions increased the enzyme activity due to its dicopper center (Fig 5).

**Fig 5:** Effect of metal ions on the polyphenol oxidase activity of Golden delicious apple fruit pulp. Each bar plot is showing the mean value of the polyphenol oxidase activity in the presence of metal ions. First bar represents mean value of the polyphenol oxidase activity in the absence of metal ions. The other three bar plots represent the polyphenol oxidase activity of apple fruit pulp in the presence of CuSO_4_, KCl, CaCl_2_. Error bars are representation of standard error (SE) of the data. Horizontal axis is showing the metal ion presence (1mM Conc) and vertical axis is showing polyphenol oxidase activity of the purified isoforms from Golden delicious apple fruit pulp.

### 3.6 PPO kinetic study

Lineweaver-Burk plot was used to find out Michaelis constant (K_m_) and maximum reaction velocity (V_max_) using catechol as substrate. K_m_ and V_max_ for apple fruit pulp PPO were found to be 74.21 mM and 4.45 μM/min (Fig 6).

**Fig 6:** Lineweaver Burk plot for the determination of K_m_ and V_max_ of polyphenol oxidase.

### 3.7 N-terminal microsequencing

Alanine residue appeared in N-terminal microsequencing of apple PPO isoform of 28 kDa molecular weight. When 28 kDa PPO band was sequenced, Alanine was the first residue followed by lysine, isoleucine, threonine, phenylalanine, histidine and glycine. The 45 kDa isoform showed alanine, proline, glycine, glycine and glycine amino acid residues (Figs 7A–7G and 8A–8E).

**Fig 7:** Graphs obtained from the applied biosystem’s pulse liquid protein sequencer. (a-g) showing the result of N-terminal microsequences (AKITFHG) of purified polyphenol oxidase isoform (28 kDa) from the fruit pulp of Golden delicious apple.

**Fig 8:** Graphs obtained from the applied biosystem’s pulse liquid protein sequencer. (a-e) showing the N**-**terminal microsequences (APGGG) of the purified polyphenol oxidase isoform (45 kDa) from fruit pulp of Golden delicious apple fruit pulp.

## 4. Discussion

The overall high yield was obtained after the purification of PPOs from Golden delicious apple fruit pulp and total yield was 27% with 6.15 folds purification. This confirms the previous finding in the literature which shows that PPOs were purified from apple using Sepharose, its specific activity after purification was calculated to be 188 μkat/mg and total yield percentage was observed as 12% [29]. Our result has significant similarity with the reported study on cashew apple where the specific activity of PPO crude extract from cashew apple was found to be 0.38 Umin^-1^mg Protein^-1^ [30]. Our findings are also consistent with the reported study on fuji apple. The specific activity of polyphenol oxidase from apple was 6800 U/mg. Purification was done with DEAE Sepharose fast slow and total PPO activity was determined to be 31410 U [31]. Two active PPO isoforms (45 and 28 kDa) were detected by SDS-PAGE in the present study. The literature on PPO purification from different plant sources shows various PPO isoforms. The existence of polyphenol oxidase isoforms has been studied previously and there were seven molecular forms of polyphenol oxidase reported in apple extract [32–34]. The differences in size and number of PPOs are due to several factors such as subcellular location of polyphenol oxidase [35], developmental stages, storage conditions [36] and artifacts formation are important [37]. Modifications of polyphenol oxidase during isolation may also occur by glycosides attachment [37]. It was found that polyphenol oxidase from apple have a carbohydrate part [38]. Artifacts generation by protease action have also been extensively reported [38]. Proteolytic process also affects the native enzyme and breaks it to several smaller active forms [39]. Modification in the protein tertiary structure of polyphenol oxidase changes the electrophoretic movement [40]. The interconversion of different forms of polyphenol oxidase has been observed during partially and fully denaturing electrophoretic condition [40, 41]. The molecular biology and genetics of polyphenol oxidase provide reasons of its existence in multiple forms. The polyphenol oxidases from different species including apple are encoded by multigene families [42, 43].

The PPO activity of Golden delicious apple fruit pulp in the given study was maximum at pH 6 and 6.5. We have found much high activity of PPO. Reported study showed that change in pH drastically effect on the polyphenol oxidase activity [44]. Similar results were also observed in recently reported research on PPO enzyme purified from banana peel and lentils [45, 46]. The available literature showed the optimum pH value of PPO from golden delicious apple to be 5.5 [47]. Our findings in the present study are in line with the reported study that shows the optimum PPO activity in jonagored apple with catechol substrate at pH 5 and 7.5. The pH 7 from sapodilla plum PPO and 6.5 (cashews apple) PPO was also observed [47–50]. Temperature optimization studies in the present work showed the highest polyphenol oxidase activity from the fruit pulp of Golden delicious apple at 40°C which decreased above that temperature. This value correlates with the reported study that confirms the optimum temperature to be 40˚C of Golden delicious apple. The maximum temperature was determined to be around 40˚C for PPO activity in many other fruits. The PPOs activity of banana pulp [51] and loquat fruit [52] is favored at 30˚C whereas at 35˚C for pear [53]. Polyphenol oxidase is an enzyme with dicopper center, so its activity was increased after the addition of copper ions. The increased in activity of PPO was reported in a study [24] in the presence of copper ions. Adding copper ions moderately activated the PPO activity of Hemsin apple [54]. K_m_ and V_max_ for apple fruit pulp polyphenol oxidase were observed to be 74.21 mM and 4.45 μM/min. K_m_ of polyphenol oxidases of different fruits vary as K_m_ from Victoria grape (52.6mM), cocord grape (67 mM), apple (230 mM) and red delicious apple (220 mM) [55–57]. When X-ray structure of PPO was studied the alanine residue appeared at the amino terminal region of the mature protein [50].

## 5. Conclusions

Our result has led us to conclude that Golden delicious apple fruit pulp contains two novel isoforms (45kDa and 28kDa) of polyphenol oxidase. The N-terminal microsequence applied for the first time to study the amino acid residues present at N-terminal. Importantly, in recent years huge information is being accumulated about various features of PPOs especially their key functions is plant physiology therefore, study and understanding the mechanism will help in the reduction of negative impact of PPO on various fruits and crops. Further, these can be used for the biological treatment of phenolic waste material to reduce environmental pollution. Possibly, our findings on the extraction, purification and characterization of PPO will be a breakthrough for its wide biotechnological applications in medicines, textile, food and paper industries. This approach can further be used in the purification of polyphenol oxidase isoforms to their crystalline structure, that can lead to better understanding of PPOs and their applications. Further research in future can be done to predict the crystalline structure of these polyphenol oxidase isoforms and their genetics can also be done to improve their activity.
